The article "Impact of Preoperative Counselling on Early Postoperative Mobilization and Its Role in Smooth Recovery" was published in 2014. Journal: Int Sch Res Notices.

# Impact of Preoperative Counselling on Early Postoperative Mobilization and Its Role in Smooth Recovery

**DOI:** 10.1155/2014/250536

**Published:** 2014-10-28

**Authors:** Sunil Sadruddin Samnani, Muhammad Farooq Umer, Syed Hussain Mehdi, Farah Naz Farid

**Affiliations:** ^1^Department of Surgery, Jinnah Medical College Hospital, S. R-6, 7/A, Korangi Industrial Area, Karachi-74900, Pakistan; ^2^Surgical Unit, Aga Khan University Hospital, Stadium Road, P.O. Box 3500, Karachi-74800, Pakistan

## Abstract

*Background and Objectives.* Preoperative counseling is effective to foster early postoperative mobilization that reduces pulmonary complications following abdominal surgery. This study aims at evaluating the effect of preoperative counseling regarding postoperative mobilization and its impact on reducing pulmonary complications. *Design and Setting.* Randomized control trial was conducted at the Department of Surgery of a tertiary care hospital, Karachi. *Patients and Materials.* Patients who underwent abdominal surgery and met inclusion criteria were recruited. All participants were randomly divided into two groups. Both groups received information about the surgery and Group I received additional counseling for postoperative mobilization. All patients were encouraged for postoperative mobilization. Scholes et al. criteria were used to evaluate postoperative pulmonary complications. *Results.* In total 232 participants were recruited and divided into two groups. There was no significant difference in participants' age (*P* = 0.79), duration of surgery (*P* = 0.5), and pain score (*P* = 0.1) of both groups. However, significant difference was identified in mobilization from bed to chair and mobilization for >10 minutes. Patients in Group I experienced less pulmonary complications in comparison with Group II.

## 1. Introduction

Postoperative pulmonary complications are found to be associated with increased morbidity and mortality following abdominal surgeries [1]. They also lead to additional health cost and prolonged length of hospital stay [2]. According to the findings reported in an Australian study, postoperative pulmonary complications are 13% prevalent and significantly prolong length of hospital stay [3]. However, various rates of pulmonary complications had been reported in the literature due to lack of proper criteria for pulmonary complications [4].

Strategies to prevent postoperative pulmonary complications have been studied at limited extent. Available evidences suggest that early postoperative mobilization following abdominal surgery contributes to improved lung volume which eventually reduces incidences of postoperative pulmonary complications [5, 6]. However, quantity of postoperative early mobilization to prevent pulmonary complication is unknown.

The article "Impact of Preoperative Counselling on Early Postoperative Mobilization and Its Role in Smooth Recovery" was published in 2014. Journal: Int Sch Res Notices.

Preoperative counseling regarding hospital stay and patient's role in recovery has proven to reduce anxiety, reduce length of stay, and have better compliance with postoperative care plan including early mobilization [7]. Eventually, preoperative counseling may contribute towards early mobilization that can reduce postoperative pulmonary complications following abdominal surgery.

Counseling regarding surgical procedures is commonly employed at every setup but less importance is given to additional counseling regarding postoperative management. This study aims at evaluating the effect of preoperative counseling regarding postoperative mobilization and its impact on reducing pulmonary complications in a developing world.

## 2. Materials and Methods

The randomized control trial was conducted at the Department of General Surgery of a tertiary care hospital of Karachi, Pakistan, from September 2012 to March 2013. Participants were recruited from outpatient clinic as well as from emergency department of the hospital. Consecutive cases were selected from the selected study setting. Study participants included patients undergoing abdominal surgery. Patients who underwent laparoscopic or minimally invasive surgeries and patients whose score was >2 on the American Society of Anesthesiologist (ASA) scale were excluded. Patients who had poor surgical outcomes and needed reexploration were also excluded from study. Moreover, patients who were smokers and had abnormal findings on X-ray were also excluded.

Patients who met the predetermined inclusion criteria were recruited in the study. Participants were divided into two groups randomly. Systemic random sampling technique was used to recruit study participants. Every second patient who visited selected study setting was recruited in Group I, whereas others were kept in Group II. Group I received informed consent regarding surgical procedure as well as counseling related to early postoperative mobilization and its impact on surgical outcome, whereas Group II received information regarding surgical procedure only. To reduce biasness, senior residents who were not part of the study conducted these counseling sessions. An information sheet was provided to patients in both English and Urdu language. Explanation was given about nature of study, rights of study participants, privacy and confidentiality of participants, and rights of withdrawal from study. Written informed consent was taken from each study participant. Study was approved by ethical committee of hospital.

Demographic and clinical information was sought from each study participant. In addition, history of previous illness, comorbidity, and any barrier to early postoperative mobilization were assessed. Both groups received counseling regarding nature of surgery and its complications, what to expect during hospitalization, postoperative pain management, and possible complications associated with surgery and anesthesia, whereas Group I received additional information regarding postoperative mobilization and its impact. All patients were given Inj. Bupivacaine locally at the time of wound closure. Patients were encouraged and assisted to mobilize once they were fully awake, with stable blood pressure and pulse, no dyspnea on rest, and pain score of <8 on Visual Analogue Scale. Data was collected preoperatively and on each day until patient gets discharged. The time at which surgery ended and the time when patient first got out of the bed (bed to chair) were recorded. In addition, time from end of surgery to first mobilization of >10 minutes was also recorded. Patients who had prolonged duration of surgery and who were smokers underwent chest physiotherapy and incentive spirometry with the help of physiotherapy staff. Postoperative pulmonary complications following abdominal surgery were assessed via criteria of Scholes et al. [3] postoperative pulmonary complications are as follows.

1. Chest X-ray showing collapsed lung or consolidation.
2. Increased body temperature >38°C for more than one consecutive postoperative day.
3. Sputum culture providing evidence of infection.
4. Productive yellow or greenish sputum.
5. Unexplained increased white blood cell count.
6. Abnormal breath sound on auscultation.
7. Diagnosis of pulmonary complication by physician.

The article "Impact of Preoperative Counselling on Early Postoperative Mobilization and Its Role in Smooth Recovery" was published in 2014. Journal: Int Sch Res Notices.

The criteria for postoperative pulmonary complications were reviewed from preoperative health status. In the current study, walk for >10 minutes was considered as early mobilization.

All gathered data were entered into SPSS version 20 for the purpose of analysis. Both descriptive and inferential analyses were conducted. *P* value of ≤0.05 was considered significant.

## 3. Results

In total, 232 patients were invited to participate in the study. They were randomly divided into two groups with 116 participants each. 2 participants in Group I and 5 participants in Group II were excluded from study because of poor surgical outcomes. 1 participant from Group I declined to continue further as part of the study because of low pain threshold. Data from 113 participants from Group I and 111 participants from Group II were analyzed. Mean age of participants in Group I was 36.70 ± 8.69 years (median: 37 years, range: 38 years) with male to female ratio of 49 : 64, whereas in Group II mean age of participants was 37.01 ± 8.43 years (median: 38 years, range 33 years) with male to female ratio of 38 : 73. There was no significant difference noted in mode of admission among these two groups (*P* = 0.43). Diagnosis of the patients and procedure performed in both groups were almost the same as shown in Table 1. Similarly, there was no significant difference in the duration of surgery (*P* = 0.51) and pain score (*P* = 0.32) among both groups. Mean duration of surgery for Group I was 64.91 mins (median: 65 mins, range: 75 mins), whereas for Group II it was 63.3 mins (median: 60 mins, range: 80 mins). Similarly, participants in Group I reported mean pain score on 3.8 (median: 5, range: 3) on given Visual Analogue Scale (VAS); however, mean pain score for participants in Group II was 3.9 (median: 4, range 5).

The article "Impact of Preoperative Counselling on Early Postoperative Mobilization and Its Role in Smooth Recovery" was published in 2014. Journal: Int Sch Res Notices.

On evaluating postoperative status of patients, significant difference was observed in participants of both groups in terms of early mobilization to bed to chair and upright mobilization for more than 10 minutes (*P* < 0.001). Patients in Group I were mobilized earlier from bed to chair (mean: 342.9 mins, median: 340 mins, and range: 105 mins) in comparison to patients in Group II (mean: 1511.1 mins, median: 1500 mins, and range: 680 mins). Likewise, patients in Group I had earlier mobilization for more than 10 minutes (mean: 360.7 mins, median: 360 mins, and range: 125 mins) in contrast to patients in Group II (mean: 1570.5 mins, median: 1570 mins, and range: 680 mins). Participants in Group I who were early mobilized had fewer pulmonary complications (7.1%) compared to Group II who had 29.7% participants suffering from pulmonary complications. As shown in Table 2, whoever fulfilled any three of the Scholes et al. [3] criteria were considered to have postoperative pulmonary complications.

On exploring the impact of counseling and support from staff for physiotherapy from Group I participants, the majority of them (68.14%) reported that counseling was very effective in providing them with motivation for early mobilization, as shown in Table 3.

## 4. Discussion

The primary aim of this study was to evaluate effect of preoperative counseling along with physiotherapy support on facilitating early mobilization among patients undergoing abdominal surgery. The study also explored impact of early mobilization on postoperative pulmonary complications.

The findings of current study revealed that early mobilization is not associated with type of abdominal surgery and its duration. Likewise, previous study has also indicated no significant difference in length of anesthesia and mobility [8].

Postoperative early mobilization in combination with physiotherapy serves as a prophylaxis to reduce postoperative pulmonary complications [8]. It has also been reported that change of position from supine to fowlers increases minute ventilation significantly [5]. Similarly, findings of current study revealed that delayed mobilization increases the risk of postoperative pulmonary complications as indicated by presence of fever, abnormal breath sounds, and cough. This finding supports that early mobilization can prevent postoperative complications associated with surgery. In line with findings of current study, early mobilization has proved to improve outcomes among patients [9–11]. Moderate level of mobility also improves muscle strength and alleviates adverse effects of immobility [12]. Hence, optimal level of mobilization is desirable among surgical patients to prevent morbidity associated with inappropriate mobilization.

The article "Impact of Preoperative Counselling on Early Postoperative Mobilization and Its Role in Smooth Recovery" was published in 2014. Journal: Int Sch Res Notices.

In the current study, patients who were mobilized earlier reported that preoperative counseling and support of physiotherapy staff were effective. In line with the current study findings, the literature revealed that increase in physical activity can be achieved among preoperative patients via continuous support [13]. Postoperative physical activity interventions have also proved to be effective in providing better surgical outcome [14, 15]. One of the study findings revealed that preoperative instructions about exercise impact postoperative compliance with exercise [16]. Such preoperative cognition interventions have proved to be effective in increasing postoperative physical activity [17]. Moreover, in developing countries where literacy level is low such interventions can significantly affect outcome of abdominal surgeries. Thus, preoperative counseling and support of physiotherapy staff can improve compliance with early mobilization which is proved to be effective in reducing postoperative pulmonary complications.

## 5. Conclusion

Early postoperative mobilization following abdominal surgery is proved to be effective in reducing pulmonary complications. In addition, preoperative counseling along with physiotherapy support can foster early mobilization among patients undergoing abdominal surgery. Hence, counseling regarding early postoperative mobilization should be promoted among patients undergoing abdominal surgery to improve surgical outcome.

## Figures and Tables

**Table 1:** Demographic and operative data.

Data	Group I (*n* = 113)	Group II (*n* = 111)	*P* value
Age (years), mean (SD)	36.70 (8.69)	37.01 (8.43)	0.79^a^
Gender, M : F	49 : 64	38 : 73	—
Mode of admission, *n* (%)			
Emergency department	62 (54.86)	55 (49.54)	0.43^b^
Outpatient department	51 (45.13)	56 (50.45)	
Diagnosis *n* (%)			
Hernia	22 (19.46)	24 (21.62)	—
Cholelithiasis/cholecystitis	41 (36.28)	35 (31.53)	
Appendicitis	25 (22.13)	28 (25.22)	
Intestinal obstruction	13 (11.5)	14 (12.61)	
Intestinal perforation	3 (2.65)	6 (5.40)	
CA colon	3 (2.65)	2 (1.80)	
Gastric carcinoma	1 (0.88)	0 ()	
Type of surgery *n* (%)			
Hernia repair	22 (19.46)	24 (21.62)	—
Cholecystectomy	43 (36.28)	35 (31.53)	
Appendectomy	25 (22.13)	28 (25.22)	
Graham's repair	1 (0.88)	5 (4.5)	
Resection and anastomosis	2 (1.76)	1 (0.9)	
Hemicolectomy	3 (2.65)	2 (1.8)	
Gastrectomy	1 (0.88)	0 ()	
Duration of surgery (mins), mean (SD)	64.91 (17.7)	63.33 (18.4)	0.51^a^
ASA score			0.32^b^
Normal	66	72	
Mild systemic diseases	47	39	
Emergency (either class I or II)	62	55	
Visual Analogue Score (VAS), mean (SD)	3.80 (0.77)	3.98 (0.92)	0.10^ a^

^a^ *t*-test for independent samples.

^b^Chi-square test.

The article "Impact of Preoperative Counselling on Early Postoperative Mobilization and Its Role in Smooth Recovery" was published in 2014. Journal: Int Sch Res Notices.

**Table 2:** Comparison of pulmonary complications.

Data	Group I (*n* = 113)	Group II (*n* = 111)	*P*-value
Mobilization (min), mean (SD)			<0.001^a^
Bed to chair	342.92 (22.93)	1511.17 (174.64)	
More than 10 minutes	360.71 (27.39)	1570.54 (170.7)	
Pulmonary complications^*^, *n* (%)	8 (7.1)	33 (29.7)	<0.001^b^
Abnormal breath sound, number (%)	9 (8)	32 (28.8)	
Fever for consecutive days, number (%)	9 (8)	8 (7.2)	
Presence of cough, number (%)	15 (13.3)	38 (34.2)	
White colored sputum, number (%)	8 (7.1)	4 (3.6)	
Yellow or green colored sputum, number (%)	3 (2.7)	34 (30.6)	
Chest X-ray showing collapse or consolidation, number (%)	5 (4.4)	30 (27)	
Unexplained rise on WBC, number (%)	2 (1.8)	5 (4.5)	

^a^ *t*-test for independent samples.

^b^chi-square test.

^*^Fulfilling criteria set by Scholes et al. [3].

**Table 3:** Impact of counseling and physiotherapy among Group I.

Data	Group I *n* (%)
Very effective	77 (68.14)
Effective	21 (18.58)
Satisfactory	11 (9.73)
Not effective	04 (3.5)

## References

[1] Warner D. O. (2000). Preventing postoperative pulmonary complications: the role of the anesthesiologist. *Anesthesiology*.

[2] Thompson D. A., Makary M. A., Dorman T., Pronovost P. J. (2006). Clinical and economic outcomes of hospital acquired pneumonia in intra-abdominal surgery patients. *Annals of Surgery*.

[3] Scholes R. L., Browning L., Sztendur E. M., Denehy L. (2009). Duration of anaesthesia, type of surgery, respiratory co-morbidity, predicted VO_2_max and smoking predict postoperative pulmonary complications after upper abdominal surgery: an observational study. *Australian Journal of Physiotherapy*.

[4] Agostini P., Naidu B., Cieslik H. (2011). Comparison of recognition tools for postoperative pulmonary complications following thoracotomy. *Physiotherapy*.

The article "Impact of Preoperative Counselling on Early Postoperative Mobilization and Its Role in Smooth Recovery" was published in 2014. Journal: Int Sch Res Notices.

[5] Zafiropoulos B., Alison J. A., McCarren B. (2004). Physiological responses to the early mobilisation of the intubated, ventilated abdominal surgery patient. *Australian Journal of Physiotherapy*.

[6] Silva Y. R., Li S. K. Developing mobility outcome measures to evaluate physiotherapy practice post abdominal surgery.

[7] Kiecolt-Glaser J. K., Page G. G., Marucha P. T., MacCallum R. C., Glaser R. (1998). Psychological influence on surgical recovery. *The American Psychologist*.

[8] Silva Y. R., Li S. K., Rickard M. J. F. X. (2013). Does the addition of deep breathing exercises to physiotherapy-directed early mobilisation alter patient outcomes following high-risk open upper abdominal surgery? Cluster randomised controlled trial. *Physiotherapy*.

[9] Morris P. E., Goad A., Thompson C. (2008). Early intensive care unit mobility therapy in the treatment of acute respiratory failure. *Critical Care Medicine*.

[10] Needham D. M., Korupolu R., Zanni J. M. (2010). Early physical medicine and rehabilitation for patients with acute respiratory failure: a quality improvement project. *Archives of Physical Medicine and Rehabilitation*.

[11] Schweickert W. D., Pohlman M. C., Pohlman A. S. (2009). Early physical and occupational therapy in mechanically ventilated, critically ill patients: a randomised controlled trial. *The Lancet*.

[12] Needham D. M. (2008). Mobilizing patients in the intensive care unit: improving neuromuscular weakness and physical function. *The Journal of the American Medical Association*.

[13] Bond D. S. (2011). Bari-active: a preoperative intervention to increase physical activity. *Obesity Surgery*.

[14] Egberts K., Brown W. A., O'Brien P. E. (2011). Optimizing lifestyle factors to achieve weight loss in surgical patients. *Surgery for Obesity and Related Diseases*.

[15] Shah M., Snell P. G., Rao S. (2011). High-volume exercise program in obese bariatric surgery patients: a randomized, controlled trial. *Obesity*.

[16] Livhits M., Mercado C., Yermilov I. (2010). Exercise following bariatric surgery: systematic review. *Obesity Surgery*.

[17] Wouters E. J., Larsen J. K., Zijlstra H., van Ramshorst B., Geenen R. (2011). Physical activity after surgery for severe obesity: the role of exercise cognitions. *Obesity Surgery*.

